# Analysis of Teaching Effect of Korean Education Course Based on Data Acquisition Technology

This article has been retracted.

**DOI:** 10.1155/2022/2541576

**Published:** 2022-08-31

**Authors:** Baoli Suo, Tao Zhang

**Affiliations:** Yantai Nanshan University, Yantai, Shandong 265713, China

## Abstract

Teaching evaluation is a comprehensive judgment of teachers' teaching effect and students' learning outcomes. It is an essential basis for comprehensive curriculum reform. There are many teaching evaluation systems for Korean majors, generally based on teachers' behavior discrimination and ignoring students' learning process and effect. The existing teaching evaluation system has problems such as heavy workload, slow calculation speed, and intense subjectivity. Based on the characteristics of Korean courses, this study constructs a teaching rating system for Korean courses in universities centered on language learning through data collection, correlation analysis, association rules, and other methods to optimize the student teaching evaluation index. At the same time, the machine learning algorithm is introduced into the teaching evaluation process to construct the teaching evaluation model and realize the automation of the teaching evaluation process. The weighted Bayesian incremental learning method is used to solve the cumulative problem of data acquisition samples. The experimental results show that the accuracy rate of classification using the weighted naive Bayesian algorithm to construct the model can reach 75%. Obviously, due to the traditional Bayesian algorithm and BP neural network algorithm, it is suitable for the teaching evaluation model of Korean majors. It provides a theoretical basis for the development of language education informatization.

## 1. Introduction

At present, the main channel of higher education is still classroom teaching. Classroom teaching is a crucial link that directly affects the quality of personnel training [1]. It is of great significance to evaluate classroom teaching. Due to the differences in cultural background and curriculum system, there are specific differences in the index system, ideas, and evaluation methods of Korean teaching evaluation in China. The main body of traditional Korean classroom teaching evaluation usually consists of experts' guidance, teachers' self-evaluation, mutual evaluation mechanism within the professional level, and students' evaluation. The role of the evaluation subject is different, and the evaluation content of each subject should also be different. However, most of the current evaluation indexes are general, and most are aimed at teachers' teaching attitudes and quality [2]. When evaluating these indexes from students' perspective, they tend to be formalized, which cannot truly reflect the advantages and disadvantages of teaching effect and cannot explain the specific factors affecting teaching effect. At the same time, analysis of the current teaching evaluation results is primarily *d* in the form of statistical reports. It is not only a heavy workload but also challenging to find hidden information in large amounts of data [3].

In recent years, the rapid development of data acquisition and data mining has gradually replaced the traditional manual data acquisition mode in education and played a significant role in education [4]. The existing data acquisition technology can quickly obtain and store data according to the requirements. In the analysis, decision-making, and storage of educational data in the later stage, the advantages of big data applications are more pronounced [5]. It has a fast calculation speed and high accuracy. Therefore, the attention to educational data collection and mining continues to increase. The output of education is the process of continuously accumulating student information. We focused on open and apparent data collection in the existing data collation and recording and the relationship between large amounts of data introduced to achieve deep-level data processing technology [6].

In foreign countries, research on educational data mining has made some progress. For example, Babié and Vekié applied the Hadoop framework to analyze student behavior by collecting data from social networks [7]. By processing the login information of students in the system, a variety of classification methods are used to analyze and predict students' behavior. Many foreign educational institutions have begun to use extensive data collection, collection, and mining technology of innovative algorithms to replace the manual data processing of traditional classroom evaluation [8]. China's colleges and universities learned from the advanced experience of foreign countries, self-made, and began to use big data-related classroom data in 2012. The data mining methods that domestic scholars use in education are association rules, decision trees, support vector machines, and so on [5]. For example, James Barker analyzed and processed students' scores and combined the Hadoop platform with the characteristics of the MapReduce programming model to improve the traditional Apriori association rule algorithm [6]. They obtained valuable information to enhance the quality of teaching.. Valuable information is obtained to guide teaching reform and improve teaching quality [9]. Arnó-Macià and Rueda-Ramos used the ID3 decision tree algorithm to mine the teaching evaluation data, obtained a relatively ideal prediction model, used the association rule algorithm to verify and compare, and analyzed the reliability of the decision tree model [10]. Data mining algorithm has been applied in education and achieved good results through continuous improvement [11].

This study evaluates the traditional classroom teaching from the perspective of students receiving Korean. The evaluation focuses on the students' learning process and uses the network of the evaluation process to replace the paper evaluation form. At the same time, the original data acquisition and data mining algorithms are improved. The purpose is to supplement the Korean teaching system. The teaching evaluation model based on the Bayesian algorithm is constructed based on the actual teaching mode. The capture of the potential law of the evaluation data is established, and the internal relations between the teaching effect and the factors affecting the teaching effect are sought. Indicators are for developing and optimizing the Korean teaching system. Finally, the purpose of rapidly and objectively evaluating the teaching effect of Korean and guiding the teaching reform is achieved. This study establishes the application system of mining technology in Korean teaching at the theoretical level. It supplements the shortcomings of the existing Korean teaching evaluation in universities and provides ideas and technical support for improving the traditional teaching model.

## 2. Data Collection and Characteristic Analysis

### 2.1. Original Data Collection

Taking the undergraduate students majoring in Korean as the research object, the teaching evaluation data of five different professional courses are collected through the network questionnaire method [12]. The original data mining is based on the evaluation results of five professional studies in Korea. The questionnaire sets 14 evaluation indicators, and all needles' proportions determine the final results. The questionnaire covers students' websites, gender, Korean course subjects, and evaluation data.  Table 1 is the original data.

### 2.2. Data Reduction and Transformation

First is data induction, attribute selection of data sets, and deleting irrelevant or redundant attributes. In other words, attributes only related to teaching effect are selected from all characteristics in the original data set to reduce the number of points considered in data mining.

Data transformation is a data form that converts original data into data that are convenient for mining. When processing the original teaching evaluation data, the descriptive language in the evaluation index—“no,” “occasionally,” “often,” and “every time”—corresponds to 1, 2, 3, and 4 assignments. In addition, because the classification algorithm used in the subsequent evaluation model construction cannot directly deal with the continuous attribute data and record the total evaluation value of the teaching effect in the form of a percentage system, it is necessary to generalize the data of percentage system and map the evaluation value to five grades: unqualified, qualified, medium, good, and excellent, which are identified by Arabic numerals 1, 2, 3, 4, and 5, respectively. The specific classification of teaching evaluation grades is shown in Table 2 .

The data converted are shown in Table 3.

The data in Table 3 correspond to 14 indicator points expressed in letters *A*–*N,* respectively, in design. The final *P* represents the total value of all indicators according to the sum of the percentage. The meaning of data is the corresponding index of all collected data, assigned according to the complementary evaluation after evaluation according to all indexes.

### 2.3. Abnormal Data Detection

The disadvantage of the Korean curriculum evaluation system is that many subjective factors may cover up the objective facts and lead to errors. It is necessary to filter data with too high skin intensity for the threshold, usually defined as data cleaning. The detection of error and abnormal data is the basis for establishing the resultant force model, which can effectively improve the calculation accuracy of the model.

In data cleaning, regression uses a function fitting data to smooth data and identify noise; the outlier detection method based on density has a good effect on outlier detection of unevenly distributed data sets.

#### 2.3.1. Multiple Linear Regression

The multiple regression analysis methods establish a prediction model through the correlation analysis of two or more independent variables and one dependent variable. When the independent and dependent variables are linear correlation, it is called multiple linear regression analysis [13].

In general, using the regression method to solve the problem includes two processes: learning and prediction. Given a training data set *T* = {(*x*_*i*_, *y*_*i*_), (*x*_*i*+1_, *y*_*i*+1_),…, (*x*_*i*+*n*_, *y*_*i*+*n*_)}, the learning process is to build a model based on training data, namely, the function *Y* = *f*(*X*); the prediction process is to determine the corresponding output *y*_*n*+1_ according to the learning model *Y* = *f*(*X*) for the new input *x*_*n*+1_ [14].

This study uses the regression method to detect the deviation of the data. The evaluation index of the standardized teaching evaluation data set uses 14 feature items as the input variable during training and the total evaluation value as the output variable during training. A prediction model is constructed to predict again the total evaluation value of all data records—the deviation between the expected value of regression and the evaluation value given by students. Given a wide range of matters, the data are used with significant variation as a candidate set of outliers.

#### 2.3.2. CLOF Outlier Detection Algorithm

In general, the predicted value obtained by the regression method will also have some errors, so if using all the data deviates from the real evaluation value for abnormal data processing, we may lose the potential weight of data. Algorithm detection using density points of deviation group: the method of the density-based local deviation group threshold detection is to set a threshold for a given data set to define the distance of any data point. If the facts in the local range are very dense, then the data point is determined as expected data points, and if the nearest point to the average data point is far away from the data point, then the data point is the outlier. The most usual method is the local outlier factor and the local. We first assign an outlier factor LOF to each data point to determine whether it is an outlier. In its region, the LOF value point depends on the density of the data. In calculating the LOF value, the specific concepts involved are defined as follows.

**Definition 1 .**

(*k* distance) In data set *D*, the *k* distance of object *P* is the maximum distance from *P* to its *k*-nearest neighbor, defined as the distance *d* (*p*, *o*) between *p* and object *o*. There are at least *k* objects in *D* whose distance to *P* is less than or equal to *P* to *o* and at most *k-1* things, whose distance to *P* is more petite than *P* to *o*.

**Definition 2 .**

(*k*-distance neighborhood) Object *P* is set as *N*_k distance_ (*P*). By setting *k* to MinPts, get *N*_MinPts_ (*P*), which includes the MinPts nearest neighbor of *P*, that is, an object that contains all *MinPts* distances not more excellent than *P*.

**Definition 3 .**

(reachable distance) Object *P* for object *o* (where *o* is the nearest points of *P*) is as follows.

**Definition 4 .**

(*P* local outlier factor) *P* is the degree of an outlier. The following formula shows

(1) $$\begin{array}{c} \text{LOF}\left(p\right)=\frac{\sum_{O\in N}\left(lrd_{MinPts}\left(o\right)/lrd_{MinPts}\left(p\right)\right)}{\left|N\left(p\right)\right|}. \end{array}$$

It can be seen from formula (1) that the higher the degree of local outlier *P* is, the greater the LOF (*p*) value is.

Based on clustering and density to improve the outlier detection algorithm, the core idea of the CLOF algorithm is carrying out *K*-means clustering first after preprocessing the original data. After clustering, the data points whose Euclidean distance from the cluster's center is less than or equal to the radius in each collection are preliminarily judged as candidate outliers. Then, for the candidate outliers, the LOF algorithm is used to detect and obtain the final outliers [15].

Among them, the *K*-means clustering algorithm is one of the most feasible and used algorithms widely in clustering analysis. The main goal is to minimize the mean square of the Euclidean distance between each element and its cluster center and divide the data set into *K* clusters with *K* as input parameters. In the process of clustering, the calculation formula of the cluster center is as follows:

(2) $$\begin{array}{c} X_{o}=\frac{\sum_{k=1}^{m}X_{k}}{n_{i}}. \end{array}$$

In the above formula, *n* is the number of data objects of class *i*, and the radius calculation formula of rank *i* is as follows:

(3) $$\begin{array}{c} R_{i}=\frac{\sum_{k=1}^{m}X_{k}-X_{o}}{n_{i}}. \end{array}$$

For each data object *X*_i_, the formula for calculating the class center *X*_o_ distance to its corresponding class is as follows:

(4) $$\begin{array}{c} d=\sqrt{\sum_{j=1}^{m}{\left(x_{ij}-x_{oj}\right)}^{2}}. \end{array}$$

The *m* in formula (4) represents the dimension of each data. The *K*-means clustering method can also detect outliers, mainly regarding the information not belonging to any class or within the course with few data objects as outliers. Still, the detection accuracy is highly dependent on the determination of clustering parameters, so the detection effect is often not pronounced [16]. CLOF has a better outlier detection effect. The steps are as follows:

  Step1: for the preprocessed data set, called the *K*-means clustering algorithm, the data set is divided into different clusters.
  Step2: the read value *m* of the number of outliers is set, and the number of data in each category *n*_i_ is counted. If *n*_i_ < = *m* determines all the data as candidate outliers, go to Step 4. If *n*_i_ > *m*, go to Step 3.
  Step3: Formulas (3) and (4) are used to calculate the class center x of each cluster. The distance di from each data point x to the center of the class is calculated by Equation (3). if *d*_i_ > = *R*, the data point is determined as a candidate outlier.
  Step4: Step 2 and Step 3 are combined to determine the candidate outliers. The LOF method calculates the outlier factor of data points for the candidate outlier set and is sorted according to the LOF value.
  Step5: the first *m* points are output with an immense LOF value, the final outlier.

The clustering process is mainly to prune the nonoutliers and obtain the candidate set of outliers to reduce the unnecessary calculation of the LOF inspection process so that analysis realizes the LOF process quickly. Therefore, the time complexity of the CLOF algorithm is significantly reduced. At the same time, because the LOF process is carried out on the candidate and selection set after pruning, the waste of space resources is avoided.

### 2.4. Feature Correlation Analysis

Without a scientific analysis and effective screening, it is difficult to ensure the independence of attributes and prone to duplication or incompleteness. Therefore, this study analyzes the correlation of the evaluation attributes designed in the questionnaire and revises the evaluation system. The correlation coefficient reflects the closeness between random variables, according to the correlation coefficient. The projects can measure the degree of correlation and interaction between attributes [17]. The following formulas show the definition.

(5) $$\begin{array}{c} r=\frac{\mathrm{cov}\left(X,Y\right)}{\sigma_{X}\sigma_{Y}}, \end{array}$$

where *r* is the correlation coefficient, representing the correlation degree of *X* and Y, and is the relative value. Cov (*X*, *Y*) is a covariance, collaborative representation data set. The larger the matter, the stronger the synergy. *σ*_*X*_*σ*_*Y*_ is the standard deviation, which is the evaluation index of data volatility. The greater the value, the stronger the volatility. For *n* different attributes, we can calculate the correlation coefficient between two so that all the correlation coefficients constitute a matrix, such as follows[18]:

(6) $$\begin{array}{c} R=\left[\begin{array}{cccc} r_{11} & r_{12} & \cdots & r_{1n}\\ r_{21} & r_{22} & \cdots & r_{2n}\\ \cdots & \cdots & \cdots & \cdots \\ r_{n1} & \cdots & \cdots & r_{nn} \end{array}\right]. \end{array}$$

The size of the correlation coefficient can indicate the degree of interdependence between the two attributes. If the correlation coefficient between the two attributes is significant, the correlation between the two attributes is strong, and if the correlation coefficient is small, the correlation is weak. Therefore, the independence between features indirectly by the value range of the correlation coefficient is analyzed.

## 3. Classroom Teaching Evaluation Model Based on Weighted Naive Bayes

This section mainly expounds on the construction process of the teaching evaluation model. Firstly, it introduces several traditional classification algorithms. Theoretical analysis and experimental verification show that adopting the Bayesian algorithm in Korean teaching is feasible. It is feasible to adopt the Bayesian algorithm in the Korean teaching mode. The weighted modification based on the traditional Bayesian algorithm can avoid the shortcomings of the conventional algorithm and establish a more targeted evaluation model for short language courses. At the same time, the weighted Bayesian classification incremental learning algorithm with improving evaluation efficiency is combined.

### 3.1. Evaluation Method Based on Traditional Classification Algorithm

There is an essential influencing factor in the learning process of the traditional model. A good supervision process must be established to summarize the typical characteristics of the data. Each classification has different modes, and the consistent model must be matched to achieve the calculation accuracy of this category. This process's summary can guide future types of collected data and automatically check them. The merge and analysis of new data by precise matching are completed, and the unclassified data are filtered and predicted. This problem includes two processes: one is autonomous learning and the other is model-based classification. The two processes are intertwined.

Machine learning under big data contains many categories. Commonly used include traditional Bayesian, support vector machine, *K*-nearest neighbor, decision tree, and neural network. The basic principles are briefly described as follows. Naive Bayes (NB) is a branch of the Bayesian theorem, which has the advantages of simple modeling, fast data processing, and rich language. The primary characteristics of data can be defined separately to avoid cross-calculation between data. The support vector machine (SVM) model belongs to binary classification. It can represent the data classifier in the spatial domain, which has a single form and is usually linear. *K*-nearest neighbor (KNN) is a fixed class decision pattern that requires only basic checking of new data and then assigning values to a specific data set. *K*-nearest neighbor algorithm is usually based on prediction and fixed label classification. The establishment of the decision tree model must cover the preprocessing and classification of the actual data and establish a tree-like system based on the generated membership characteristic degree distribution. Different branches of the tree are given utterly other category characteristics. The artificial neural network is entirely different from the above single linear model, which can deal with nonlinear data relations, especially for mining and processing confidential data and classifying chaotic data sets.

The evaluation of Korean teaching should be combined with expert opinions, teachers, and students' rating content. When selecting the evaluation model, different opinions are defined as input data, and the feature fusion of the model is as follows:

(7) $$\begin{array}{c} \text{pre}\_\text{rate}=\frac{N_{c}}{N}. \end{array}$$

This study uses different classifiers for the test process, and all the data are compared and analyzed. The selected training data adopt fixed parameters and formulas (7). The training steps and process of the calculation model are the same. For the 400 data of the students in our school, more than 30 times of cross-analysis are carried out. Finally, the experimental results of the accuracy of various classifiers are obtained.

According to the experimental data in Table 4, the average classification accuracy of these classification algorithms is compared busing the teaching evaluation data set, as shown in Figure 1.

For the same experimental data set, the average time consumption of each algorithm is shown in Table 5.

Table 5 shows that the traditional Bayesian algorithm is the best model for Korean teaching evaluation. Its advantages are high accuracy and fast calculation speed. The Korean professional curriculum evaluation model constructed in this study is based on the improvement of the traditional Bayesian model.

### 3.2. Principle of Naive Bayes Algorithm

Bayesian classification 2 is a classification algorithm based on the Bayesian theorem. The basic principle of classification is to obtain the prior probability of each category by learning a large number of training data, and then, the posterior probability of an instance *X* belonging to different types is calculated. Finally, the instance as a class with the maximum posterior probability is determined. Suppose *D* is the training data set, *A*={*A*_1_, *A*_2_,…, *A*_*n*_} is the attribute variable set, and *n* is the number of attributes. *C*={*C*_1_, *C*_2_,…, *C*_*m*_} is the set of class variables, and *m* is the number of classes, which express a training sample as {*x*_1_, *x*_2_,…, *X*_*n*_, *C*_*j*_},  *j* ∈ *m*, *C*_*j*_; say, a test sample *X* as {*x*_1_, *x*_2_,…, *x*_*n*_} is known. The probability of the test sample belonging to a specific class is judged; the following formula shows the calculation formula.

(8) $$\begin{array}{c} p\left(C_{j}|X\right)=\underset{C_{j}}{\arg\max}\frac{p\left(X|C_{j}\right)p\left(C_{j}\right)}{p\left(X\right)}. \end{array}$$

The naive Bayesian model adopts the network structure shown in Figure 2: the advantages of the model are short calculation path, high calculation efficiency, and simple calculation process.

Figure 2 shows the basic linear structure, and the centralized node is defined as the classification variable, represented by the letter *C*. The branch node is defined as the membership variable, which *A*_*i*_ characterizes. Based on the traditional Bayesian model, this model unifies all the membership degrees into class variables to eliminate the uniqueness of the original model. The calculation process can be defined as a constant *P*, and the algorithm can be implemented by the following formula:

(9) $$\begin{array}{c} p\left(C_{s}|X\right)\propto \underset{C_{s}}{\arg\max}p\left(X|C_{s}\right)p\left(C_{s}\right), \end{array}$$

where *p* (*C*_s_) is the class prior probability, which is obtained by learning the training data. The calculation formula is as follows:

(10) $$\begin{array}{c} p\left(C_{s}\right)=\frac{s_{s}}{s}, \end{array}$$

where *s*_s_ represents the number of class *C*_s_ in the training samples, and *s* represents the total number of training samples.

NB algorithm ignores the relationship between variables, assuming that the conditions between membership are independent without the cross. Based on this assumption, each variable can be classified by *C*. If the content of the data set is less than the total amount of data, it will lead to too many categories can not being labeled, the calculation process will become too cumbersome, and calculation and training time increase. Ignoring the correlation between data can effectively avoid such problems, but the corresponding calculation accuracy will decrease slightly. The calculation formula after missing the correlation is as follows:

(11) $$\begin{array}{c} p\left(X|C_{s}\right)=\prod_{i=1}^{n}p\left|x_{i}|C_{s}\right|, \end{array}$$

where *p*(*x*_1_*|C*_*s*_), *p*(*x*_2_*|C*_*s*_),…, *p*(*x*_*n*_*|C*_*s*_) learns from training data. Combined with the above three equations, the category of test data can be determined.

The traditional Bayesian algorithm assignment correlation is canceled. Its intrinsic meaning is to weaken the original characteristics of the strength of the relationship between the impacts of attributes into no difference. In an actual assignment, the weight of feature extraction must be different, so given the exact constant cause, the calculation accuracy is lower than the traditional Bayesian algorithm.

Because of the above problems, this study distinguishes the classification attributes based on the traditional Bayesian algorithm. The weight is determined according to the contribution of different characteristics, and the defined weight is given different values in the calculation. The test verifies that this method can not only meet the calculation speed of the traditional model but also significantly improve the actuarial accuracy. For the calculation process, see the following formula.

(12) $$\begin{array}{c} p\left(C_{s}|X\right)=\arg\max p\left(C_{s}\right)=\prod_{i=1}^{n}p{\left(A_{i}|C_{s}\right)}^{w_{i}}. \end{array}$$

The *A*_*i*_ particular threshold in the formula is assigned to different weights to reflect the importance of values in independent eigenvalues. There is a big difference in Korean teaching evaluation data sources, and the traditional Bayesian formula cannot skip this difference. This paper's new weighted Bayesian model can correlate the correlation between different indicators. Each attribute is defined as *A*_*i*_. The advantage of a class function is that a single-class function can still contain multiple other domains, and the formula is reflected in the difference in the *k* value. The new model in this study uses *a*_*k*_ to represent different values in the definition domain, *k* ∈ *K*. It is assumed that there is a fixed attribute Ai of *X*, and the importance of Ai of *X* is *a*_*k*_. The calculation formulas of the correlation probability *p*(*A*_*i*_*|rel*) and the uncorrelated probability *p*(*A*_*i*_*|*norel) of *A* concerning *C*_j_ in the category set are as follows:

(13) $$\begin{array}{c} p\left(A_{i}|\text{rel}\right)=\frac{\text{count}\left(A_{i}=a_{k}\wedge C_{j}\right)}{\text{count}\left(A_{i}=a_{k}\right)}, \end{array}$$

where count represents the statistics. When the value of attribute *A*_*i*_ is *a*_*k*_ and belongs to *C*_*j*_, the calculation formula of attribute weight is as follows:

(14) $$\begin{array}{c} w\left(A_{i},a_{k},j\right)=\frac{p\left(A_{i}|\text{rel}\right)}{p\left(A_{i}|\text{norel}\right)}. \end{array}$$

Therefore, the specific formula of weighted naive Bayes classification algorithm is as follows:

(15) $$\begin{array}{c} p\left(C_{j}|X\right)=\underset{C_{j}}{\arg\max}p\left(C_{j}\right)\prod_{i=1}^{n}p{\left(A_{i}|C_{j}\right)}^{w\left(A_{i},a_{k},j\right)}. \end{array}$$

The data set *D* of membership degree has *m* subsets, and *n* membership degrees can be defined. Taking *k* as the possible number of values, the membership degree of all deals is synthesized as *m∗n∗k*. Weight is based on different assignments to distinguish its importance. Other values for other classes can also be assigned to each independent category. The model automatically matches the verified labels in all labels to complete the calculation. The calculation results are reflected in the form of probability. Significant probability indicates a high weight of classification results. The weighted process is the process of training a large number of data calculations. According to the above case, the total data *D* are divided into *m* subsets, and *n* characteristic functions with the same membership degree are completed. The complete calculation results are still *m∗n∗k*. The specific steps are as follows.

  Input: examples to be classified are tested.
  Step1: all the data samples are collected as the sample set, the number of class labels Ci is counted, and the number of models whose attribute *A*_*j*_ is *a*_*k*_ is counted, and the number of samples whose attribute *A*_*j*_ is not *a*_*k*_ is recorded in the count table.
  Step2: learning-related probability parameters. According to the data in the count table, the correlation probability and non-correlation probability of all attribute values are calculated by formulas (14) and (15), and the results are saved in the RP table.
  Step3: learning weight parameters. The membership of all data in the RP table is calculated, and the corresponding label items are automatically matched. According to the label assignment matching weight, the calculation results are saved in the weight table.
  Step4: learning prior probability. According to the matching existing bibliographic synthesis, combined with formula (10) to calculate the likelihood of all types of files, the folder CPT is saved.
  Step5: The label of membership degree is self-trained. After all the data are classified and saved, the prior probability table CP and the probability table CPT are used to divide the subset further. Specific sub-data sets correspond to weight probability by weight percentage. Quotation (12) accurately calculates the probability distribution and outputs the results according to the output weights.

## 4. Evaluation Results and Analysis

### 4.1. Data Collection

#### 4.1.1. Questionnaire Design

This study expands students' evaluation of teaching for Korean learners. A network questionnaire of classroom teaching evaluation from two aspects of teachers' teaching and students' learning behavior is formed. Among them, the assessment of teachers' teaching behavior mainly includes seven indexes, including classroom teaching atmosphere, homework requirements and guidance, and teaching content extension. Students' learning behavior evaluation also contains seven indicators, including learning initiative, awareness of cooperation and communication, learning seriousness, and other aspects of assessment [19].

We combine teaching and learning behavior, and the evaluation system has 14 indexes. Most of the indexes have four evaluation results for selection, namely, no, occasionally, often, and every time. Students can give evaluation results for each index according to the teaching situation. Finally, students should provide the total evaluation value of teaching in a percentage system as the final evaluation of the teaching effect.

The experimental environment is the Windows10 operating system. python3.5 is used as the algorithm to realize the specific calculation on the Eclipse + Pydev experimental platform.

Experiment 1: comparison of classification accuracy between NB and WNB.

Four hundred experimental data were collected from the Korean students' evaluation database. The results of Table 6 are calculated by the NB algorithm and WNB algorithm with the exact definition and parameters. The results show the calculation accuracy of different algorithms.

From Table 6, Figure 3 shows the comparison of classification accuracy between the NB algorithm and WNB algorithm.

The results in Table 6 show that the accuracy of the two algorithms is different, and the average value of weighted Bayesian is higher than that of the standard algorithm. This conclusion can prove that the revised calculation model in this study has higher accuracy in the calculation results of teaching evaluation for Korean majors. It is a more suitable calculation model.

Experiment 2: comparison of classification accuracy between BP and WNB.

BP neural network is one of the most mature algorithms used in teaching data calculation. This study compares the model constructed for evaluating the teaching effect of Korean majors with the BP method, and the analysis results have guiding significance for further improvement of the model.

BP neural network normalizes all the data information of mobile phones, especially many details of different orders of magnitude. The normalization process is the process of training new simulation samples. Usually, there is a significant error in this process. In this study, aiming at the error problem of the BP neural network, the test set is added to the database training set of the traditional model. The following parameter environment is set: input layer defined as 20, hidden node and output node defined as 5, using the ( ) activation function, learning rate is 0.001, and the number of cycles is 20000.

After neural network algorithm training, the test results are shown in Table 7.

According to the data analysis of all the experimental results, because in the actual evaluation process, the percentage system evaluation value given by students is generally high, so in the model training process, it is accessible to overfit, resulting in naturally high prediction level. Therefore, considering the use of pretreatment, the percentile score value is discretized into the five-level evaluation value, and randomly selected different levels of data are mixed into training data sets, including 220 data in the training set and 70 data in the test set. A cross-experimental comparison of the BP network and WNB algorithm is carried out. The experimental results are shown in Table 8 and Figure 4.

From Table 8, the comparison of classification accuracy between NB algorithm and WNB algorithm is shown in Figure 4.

It can be seen from the diagram that the data set for all evaluations of Korean majors can be collected according to the requirements. The rating results show that excellence accounts for the highest proportion. This is consistent with the results of traditional evaluation methods. The average accuracy of the WNB algorithm is 0.74, the accuracy of the BP algorithm for the same data sample is 0.67, and the accuracy is improved by 10.4%. This paper's calculation effect of the modified weighted Bayesian algorithm is obviously due to the BP algorithm. Compared with the calculation time of the two algorithms, WNB consumes less time than the BP algorithm, and the improved algorithm is more concise. It has been proved that the modified algorithm is suitable for the teaching evaluation of Korean majors and is a calculation method worthy of promotion.

## 5. Conclusion

This study uses data analysis and modeling analysis based on data mining techniques and machine learning methods. Because of the shortcomings of the teaching evaluation system in the traditional Korean classroom, the classification algorithm of model construction is modified to further improve the scientificity and feasibility of teaching evaluation. The main achievements of this study are as follows:

1. Data mining technology is used to preprocess the obtained Korean professional classroom teaching data and an outlier detection algorithm to clean the data. Using correlation coefficients, association rules, and other methods to determine indicators' independence improves teaching evaluation's efficiency.
2. The classification algorithm in machine learning is introduced to construct the teaching evaluation model, and the weighted naive Bayesian algorithm is proposed to design the classifier. Through a large number of data training, the corresponding weights are given to each evaluation index, proving that the weighted naive Bayesian algorithm is more suitable for classroom teaching evaluation of Korean majors than the traditional BP neural network algorithm.
3. Weighted Bayesian incremental learning method is used to solve the problem of rapid data growth. The model parameters are constantly updated according to the new sample data, which improves the algorithm's efficiency and saves the data calculation time. The experimental results show that the incremental learning method can improve the time efficiency of the big data teaching evaluation scale.

## Figures and Tables

**Figure 1:** Comparison of average classification accuracy of common algorithms.

**Figure 2:** Model of naive Bayes classification.

**Figure 3:** Comparison of classification accuracy between NB algorithm and WNB algorithm.

**Figure 4:** Comparison of classification accuracy between BP algorithm and WNB algorithm.

**Table 1:** Partial raw data.

Number	IP	Time	Evaluation of subjects	Gender	Index 1	…	Index 14	Comprehensive assessment
1	138.531.	2022.3.16	Korean grammar	Female	Occasionally	…	Occasionally	100
2	117.012	2022.3.16	Korean writing	Female	Often	…	Occasionally	83
3	179.365	2022.3.16	Korean audiovisual speaking	Female	Often	…	Often	77
4	306.291	2022.3.16	Form and policy	Male	Occasionally	…	Occasionally	98
5	121.718	2022.3.16	Basic Korean	Female	Occasionally	…	Often	92

**Table 2:** Corresponding system of evaluation index.

QoS class identifier	Percentage	Hierarchy
5	90–100	Excellent
4	80–90	Fine
3	70–80	Medium
2	60–70	Qualified
1	<60	Disqualification

**Table 3:** Part of the processed data set.

Characteristic item	*A*	*B*	*C*	*D*	*E*	*F*	…	*M*	*N*	*P*
5	3	4	4	4	4	4	…	4	4	5
4	3	4	4	3	3	3	…	3	3	4
3	2	2	4	4	4	4	…	4	2	5
2	2	3	2	3	3	3	…	2	2	5
1	2	4	2	2	2	2	…	2	2	4

**Table 4:** Table of classification accuracy.

Algorithm	1	2	3	4	5	6	7	8	9	10	Mean value
NB	0.8	0.75	0.8	0.74	0.75	0.8	0.75	0.72	0.72	0.77	0.76
SVM	0.67	0.58	0.67	0.75	0.75	0.72	0.71	0.65	0.74	0.71	0.69
KNN	0.68	0.75	0.67	0.74	0.67	0.68	0.68	0.67	0.74	0.68	0.70
DT	0.65	0.62	0.68	0.7	0.64	0.71	0.72	0.65	0.70	0.65	0.67
BP	0.79	0.77	0.79	0.81	0.72	0.71	0.74	0.66	0.72	0.72	0.72

**Table 5:** Table of average running time(unit:s).

Algorithm	NB	SVM	KNN	DT	BP
Average time	0.06	28.96	3.35	0.13	34.90

**Table 6:** Classification accuracy of NB and WNB.

Algorithm	1	2	3	4	5	6	7	8	9	10	Mean value
NB	0.72	0.70	0.71	0.67	0.70	0.71	0.72	0.75	0.72	0.68	0.71
WNB	0.70	0.75	0.77	0.729	0.78	0.72	0.84	0.74	0.70	0.72	0.75

**Table 7:** Partial experimental results of BP algorithm.

Real evaluation value	Characteristic value	Predictive value	Error range	Prediction grade
0.92	Excellent	0.95	0.065	Excellent
0.95	Excellent	0.92	0.033	Excellent
1	Excellent	0.97	0.077	Excellent
0.92	Excellent	0.91	0.051	Excellent
0.97	Excellent	0.99	0.044	Excellent
0.91	Excellent	0.94	0.031	Excellent
1	Excellent	0.92	0.081	Excellent
0.89	Good	0.93	−0.091	Excellent
0.53	Below proof	0.82	−0.234	Good
0	Below proof	0.28	−0.271	Below proof

**Table 8:** Classification accuracy of BP algorithm and WNB algorithm.

Algorithm	1	2	3	4	5	6	7	8	9	10	Mean value
BP	0.74	0.65	0.67	0.62	0.77	0.65	0.70	0.729	0.64	0.62	0.67
WNB	0.72	0.78	0.81	0.72	0.75	0.77	0.72	0.84	0.72	0.78	0.74

## Data Availability

The data set can be accessed upon request.
